# Reynolds-average Navier-Stokes turbulence models assessment: A case study of CH_4_/H_2_/N_2_-air reacting jet

**DOI:** 10.1016/j.heliyon.2024.e26956

**Published:** 2024-03-06

**Authors:** Yaniel Garcia Lovella, Idalberto Herrera Moya, Jeevan Jayasuriya, Julien Blondeau

**Affiliations:** a Universidad Central “Marta Abreu” de Las Villas, Faculty of Mechanical and Industrial Engineering, Center for Energy and Environmental Technology Assessment, Santa Clara, 50100, Cuba; b Royal Institute of Technology, Department of Energy Technology, Stockholm, 10044, Sweden; c Vrije Universiteit Brussel, Faculty of Engineering, Thermo and Fluid Dynamics, Brussels, 1050, Belgium; d Vrije Universiteit Brussel (VUB) and Université Libre de Bruxelles (ULB), Brussels Institute for Thermal-Fluid Systems and Clean Energy (BRITE), Brussels, 1050, Belgium

**Keywords:** Turbulence modelling, Turbulence-chemistry interaction, Reacting jet, Jet's spreading rate

## Abstract

Computational Fluid Dynamics has become a very powerful tool for developing engineering combustion devices, such as burners and furnaces. However, there are a wide variety of turbulence models, and some of them have proven to be more effective for some turbulent flow configurations than others. A reacting turbulent jet is a common flow configuration found in combustion engineering devices like burners. The present work assesses Reynolds-Average Navier-Stokes turbulence models, being tested on a CH_4_/H_2_/N_2_-Air reacting jet. Eight two-equation eddy-viscosity and three five-equation turbulence models were tested in the studied turbulent flow. Computational results were compared against experimental measurements in terms of flow field variables, mean mixture fraction, temperature, and species mass fraction. The findings suggest a strong influence of the turbulence model perforce on the mean mixture fraction as well as on the turbulence-chemistry interaction model. The modified version of the standard k-ε model proves to be the more reliable choice for this reactive flow configurations. Specially, where the flow patterns of the jet dictate the general flow physics. Near the fuel nozzle, both the Reynolds stress model with stress baseline k-ω (RSM-SBSL) and the standard k-ω model exhibit better agreement with experimental data than the conventional modified k-ε model. Moreover, findings from the standard modified k-ε model indicate a significant underestimation of spreading rates for radial samples in regions where jet spreading intensifies.

## 1 Introduction

The importance of the combustion process in modern society has led to considerable progress in such matters. The improvements achieved in the last few decades regarding combustion science have made engineers capable of designing more demanding mechanical devices for transforming chemical energy into heat and power [1]. Traditionally, combustion studies have been addressed experimentally and are barely supported by computational techniques. In recent decades, the development of High-Performance Computing (HPC) and Computational Fluid Dynamics (CFD) has allowed powered experimental studies with analytic-numeric models [2].

The mixing process of fuel and oxidizer streams is a key factor for an efficient combustion process. Gas combustion is a common engineering application, in which is desired turbulent flow regime, considering the slow reactants mixing process under laminar reacting flows [3,4]. Turbulent flow is characterized by intense exchanges of heat, mass and momentum. However, the mixing process is strongly related to the motion structures. Large eddies are responsible for the global fluid motion and small eddies are responsible for the molecular transport and some of the small eddies fall into the mixing range. However, a zone occupied by a large eddy could contain small eddies as well, meaning that different time and length scales of motion coexist [[5], [6], [7]]. The coexistence of different eddy sizes makes turbulence modelling challenging, but important for estimating the mixing rate of fuel and oxidizer streams during the combustion process [8].

Turbulence modelling is addressed from three main approaches: Direct Numerical Simulation (DNS), Large Eddy Simulation (LES) and Reynolds-Average Navier-Stokers (RANS) [6,9]. DNS is out of reach in engineering applications, only small domains with moderated Reynolds numbers have been successfully simulated using this approach [[10], [11], [12]]. LES is a trade-off between DNS and RANS models, in terms of accuracy and computational cost. The implementation of LES modelling approach to industrial applications is still restricted by the high computational cost [13]. RANS models are less computationally expensive, but small and large eddy scales are not resolved. RANS models show a simplified representation of a very complex reality taking place under turbulence scales, which is based on Kolmogorov hypotheses and the Boussinesq turbulent viscosity approximation for estimating Reynolds stress term [14]. RANS models have become a powerful tool for dealing with turbulence modelling for industrial applications. However, about a dozen of RANS models have been developed with different formulations for estimating Reynolds Stress term [15]. Reynolds Stress computation is strongly based on empirical knowledge, which has been built under specific experimental conditions [5]. Furthermore, how well a particular RANS turbulent model fits real conditions matters for selecting the right model.

The main purpose of the present work is to assess different RANS models capability for a reacting jet flow and investigate the influence of flow field variables in the combustion chemistry. Simulation results will be compared with experimental data, providing insights regarding RANS models and steady diffusion-flamelet model capability for turbulence and combustion chemistry interaction for reacting gas jets. The experimental data used for assessing the performance of turbulence were taken from the International Workshop on Measurement and Computation of Turbulent Flames (TNF Workshop) [[16], [17], [18]].

## 2 Background

### 2.1 Governing equations for reactive fluid flow

Equations (1), (2), (3) show density-weighted averaging governing equation for fluid flow. However, density change by pressure is neglected and density changes by temperature is considered through ideal gas state model [[10], [11], [12],^19^].

(1) $$\frac{\partial \bar{\rho }}{\partial t}+\frac{\partial }{\partial x_{i}}\left(\bar{\rho }{\tilde{u}}_{i}\right)=0$$

(2) $$\frac{\partial \bar{\rho }{\tilde{u}}_{i}}{\partial t}+\frac{\partial }{\partial x_{j}}\left(\bar{\rho }{\tilde{u}}_{i}{\tilde{u}}_{j}\right)+\frac{\partial \bar{p}}{\partial x_{i}}=\frac{\partial }{\partial x_{j}}\left({\bar{\tau }}_{\text{ij}}-\bar{\rho u_{i}^{\prime \prime }u_{j}^{\prime \prime }}\right)$$

u represents the three velocity components, ρ is the density, τ is the viscous stress tensor, t is the time and x represents the three coordinated directions.

The Reynolds stresses term in Eq. (2) $\left(-\bar{\rho u_{i}^{\prime \prime }u_{j}^{\prime \prime }}\right)$ will be the object of further analysis, if it is considered that closure models should be provided for dealing with such term. Eq. (3) represents the energy transport equation for a multi-species gas mixture, considering a single diffusion coefficient for all species and Lewis number equal to unit. $\left({\bar{S}}_{h}\right)$ represents the energy source term, which account for all energy contributions per unit of volume defined as a source, including radiation contribution $\left({\bar{S}}_{h,\text{rad}}\right)$.

(3) $$\frac{\partial }{\partial x}\left(\bar{\rho }\tilde{h}\right)+\frac{\partial }{\partial x_{j}}\left(\bar{\rho }{\tilde{u}}_{j}\tilde{h}\right)=\frac{\partial }{\partial x_{j}}\left(\Gamma_{h}\frac{\partial \tilde{h}}{\partial x_{j}}\right)+{\bar{S}}_{h}$$

Energy equation is formulated as function of enthalpy (h). ${\;\Gamma }_{h}=\left(\mu /\sigma +\mu_{t}/\sigma_{h}\right)$, $\mu_{t}$ is the turbulent viscosity and $\sigma_{h}$ is the turbulent Prandtl number. The contribution of radiative heat transfer to the source terms of the energy equation is depicted as shown in Eq. (4).

(4) $${\bar{S}}_{h,\text{rad}}=\frac{1}{\Delta V}\int q_{\text{rad}}∙ndA=\frac{1}{\Delta V}\int \left(q_{-}-q_{+}\right)dA$$

The net radiative heat flux $\left(q_{\text{rad}}\right)$ is computed from the incident radiative flux $\left(q_{-}\right)$ and the outgoing radiative flux $\left(q_{+}\right)$. The incident and outgoing radiation fluxes are determined based on the intensity of the radiative fluxes (I). Eq. (5) is known as Radiative Transfer Equation (RTE), used to compute radiative flux intensity.

(5) $$\frac{dI\left(\vec{x},\vec{s}\right)}{ds}+\left(a+\sigma_{s}\right)I\left(\vec{x},\vec{s}\right)={an}^{2}\frac{\sigma T^{4}}{\pi }+\frac{\sigma_{s}}{4\pi }\int_{0}^{4\pi }I\left(\vec{x},\vec{s}\right)\Phi \left(\vec{x},\vec{s}\right)\;d\Omega$$

In Eq. (5), the computed radiation intensity $I\left(\vec{x},\vec{s}\right)$ is determined, considering the direction $\left(\vec{s}\right)$ at each position $\left(\vec{x}\right)$. Given the absence of solid particles during gas combustion, the absorption coefficient of flue gas $\left(\sigma_{s}\right)$ and refractive index (n) are set to one and $0s^{-1}$, respectively. Here, Φ represents the phase function, Ω denotes the solid angle, and a stands for the scattering coefficient. Therefore, a simplified model, known as the Discrete Ordinaries (DO) model, was selected for computing I in the conducted study [20,21].

### 2.2 Turbulence and chemistry interaction modelling

The interaction between turbulence and chemistry is based on the modelling approach originally proposed by Peters [22]. The steady laminar flamelet model relies on the concept of treating a turbulent flame as an assembly of laminar diffusion 1D-flames, called flamelets. The moving laminar parcel of reactive flow (a single flamelet) reacts and releases most of the heat in the vicinity of the stoichiometric contour of the flame. Nevertheless, a real turbulent flame, which is represented in the model as the entire assembly of laminar flamelets, is constantly stretched and strained by the flow turbulence. The model is implemented in three major steps: 1) the generation of laminar flamelet libraries, 2) the computation of Favre-averaged values of scalar quantities in the turbulent flow field and 3) the computation of the mean mixture fraction, it variance and scalar dissipation rate during CFD calculation as field variable [23].

In the first step, the thermochemical state of gas mixture is related to a conserved scalar quantity called mixture fraction (ξ), see Eq. (6). $Z_{i}$ is the elemental mass fraction of element i, $Z_{i,\text{ox}}$ is the elemental mass fraction of element i at the inlet of oxidizer stream and $Z_{i,\text{fuel}}$ is the elemental mass fraction of element i at inlet of the fuel stream.

(6) $$\xi =\frac{Z_{i}-Z_{i,\text{ox}}}{Z_{i,\text{fuel}}-Z_{i,\text{ox}}}$$

The chemistry of the combustion process is assumed to be represented by the governing equations of opposed flow diffusion flames, which are transformed into mixture fraction space, as shown in Eq. (7) and Eq. (8) (Flamelet equations). The formulation of Eq. (7) and Eq. (8) assumes that Lewis number is equal to unit.

(7) $$\rho \frac{\partial Y_{k}}{\partial t}+\rho \frac{x}{2}\frac{\partial^{2}Y_{k}}{\partial \xi^{2}}-{\dot{\omega }}_{k}=0$$

(8) $$\rho \frac{\partial T}{\partial t}+\rho \frac{x}{2}\frac{\partial^{2}T}{\partial \xi^{2}}-\frac{1}{C_{p}}\frac{\partial p}{\partial t}{+\sum_{k=1}^{N}\frac{h_{k}}{C_{p}}\dot{\omega }}_{k}=0$$

The steady-state solution of flamelet equations is obtained by solving Eq. (7) and Eq. (8) for specific boundary conditions, for the fuel stream $\left(\xi =1:{T=T}_{\text{fuel}}\;{\;Y}_{k}={\;Y}_{k,\text{fuel}}\;k=1,\ldots ,N\right)$ and for the oxidizer stream $\left(\xi =0:{T=T}_{\text{oxidizer}}\;{\;Y}_{k}={\;Y}_{k,\text{oxidiser}}\;k=1,\ldots ,N\right)$ and within a given range of scalar dissipation rate. The solution of flamelet equations requires a chemical mechanism to compute the reaction rate of each species during each considered reaction. In the step of generating the laminar flamelet library, chemistry is assumed to control the described physics of the flame at this point in the model. Therefore, elaborate chemistry can be economically incorporated to generate density, temperature, and species mass fraction profiles [12]. In the present study, the GRI-MECH 3.0 chemical mechanism [24] is used, consisting of 325 reactions and 53 species. This mechanism has been successfully implemented with the steady laminar flamelet model in combustion applications involving methane blends for RANS simulations [[25], [26], [27]].

In the second step, the Favre-averaged values of scalar quantities in the turbulent flow field are computed. The influence of turbulence fluctuations on the thermochemical state of the flame is a key factor to consider for achieving a realistic representation of turbulent flames. The Jones and Whitelaw principle provide a solution to compute the density-weighted average of an arbitrary scalar quantity $\left({\tilde{\varphi }}_{i}\right)$, see Eq. (9) [28].

(9) $${\tilde{\varphi }}_{i}=\iint \varphi \left(\xi ,x_{\text{st}}\right)\tilde{P}\left(\xi ,x_{\text{st}}\right)d\xi dx_{\text{st}}$$

β-probability density function (pdf) is assumed for the definition shown in Eq. (9). Then, Favre mean density, species concentration and enthalpies $\left({\tilde{\varphi }}_{i}\right)$ are tabulated as a function of mixture fraction $\left(\tilde{\xi }\right)$, its variance $\left({\tilde{\xi }}^{\prime \prime 2}\right)$ and scalar dissipation $\left(x_{\text{st}}\right)$. In a few words, pdf could be addressed as the fraction of time in which gas mixture will be at state ξ.

In the third step, the CFD model solves the Favre mixture fraction equation (Eq. (10)) and its variance (Eq. (11)), simultaneously with fluid flow, energy, and RTE equations.

(10) $$\frac{\partial }{\partial t}\left(\bar{\rho }\tilde{\xi }\right)+\frac{\partial }{\partial x_{j}}\left(\bar{\rho }{\tilde{u}}_{j}\tilde{\xi }\right)=\frac{\partial }{\partial x_{j}}\left(\Gamma_{\xi }\frac{\partial \tilde{\xi }}{\partial x_{j}}\right)$$

(11) $$\frac{\partial }{\partial t}\left(\bar{\rho }{\tilde{\xi }}^{\prime \prime 2}\right)+\frac{\partial }{\partial x_{j}}\left(\bar{\rho }{\tilde{u}}_{j}{\tilde{\xi }}^{\prime \prime 2}\right)=\frac{\partial }{\partial x_{j}}\left(\Gamma_{\xi }\frac{\partial {\tilde{\xi }}^{\prime \prime 2}}{\partial x_{j}}\right)+C_{g1}\mu_{t}∙{\left(\frac{\partial {\tilde{\xi }}^{\prime \prime 2}}{\partial x_{j}}\right)}^{2}-C_{g2}\rho \frac{\tilde{\varepsilon }}{\tilde{k}}\rho {\tilde{\xi }}^{\prime \prime 2}\text{,}$$

In Eq. (9), $\Gamma_{\xi }=\left(\mu /\sigma +\mu_{t}/\sigma_{\xi }\right)$, where $\sigma_{\xi }$ is represents the turbulent Schmidt number. Additionally, in the Favre-averaged mixture fraction variance $C_{g1}$ and $C_{g2}$ are model dimensionless constant with values of 2.0 and 2.8, respectively. The influence of the mixture fraction distribution on the fluid flow field to the thermochemical state is considered by the scalar dissipation rate, as Eq. (11) shows.

(12) $$x=2D_{\xi }\left[{\left(\frac{\partial \xi }{\partial x}\right)}^{2}+{\left(\frac{\partial \xi }{\partial y}\right)}^{2}+{\left(\frac{\partial \xi }{\partial z}\right)}^{2}\right]\text{,}$$

In Eq. (12), $D_{\xi }=\Gamma_{\xi }/\rho$, where $D_{\xi }$ represents the diffusion coefficient of the mixture fraction. The CFD model computes the distribution of the mean mixture fraction, its variance, and the scalar dissipation rate in the flow field. Subsequently, the Favre-averaged values for density, temperature, and species mass fraction are obtained from precomputed steady laminar flamelet libraries. This approach allows users to reduce the computation of combustion chemistry during CFD calculations to three scalar quantities. Meanwhile, the chemistry is pre-processed before CFD calculation begins. The relatively low computational cost associated with handling combustion chemistry in the steady laminar flamelets model encourages the implementation of elaborate chemical mechanisms. However, it is worth noting that the flame reacts quickly to changes in the scalar dissipation rate parameter for turbulent flames, making flow time scales the limiting quantity on the combustion process instead of chemical time scales. The model is considered under the assumption of fast chemistry [29]. Nevertheless, it is also regarded as a compromise between simplicity and the need to account for detailed chemistry [12]. Therefore, effects far from equilibrium, such as flame lift-off, ignition delay, and local extinction, could be more challenging to assess using this combustion modelling approach [12,19,29].

### 2.3 Turbulence models assessment

RANS turbulence models deal with Reynolds stresses $\left(-\bar{\rho u_{i}^{\prime \prime }u_{j}^{\prime \prime }}\right)$ to provide new closure equations [5,9,12]. These models are classified based on the number of additional transport equations needed to be solved along with fluid flow, energy, and any other scalar equations.

The zero-equation model, known as Prandtl's mixing length model is the most validated turbulence model. However, like the one equation model presented by Spalart and Allmaras [30], those models offer limited information about the flow field, resulting in quite inadequate links to the steady diffusion-flamelet model. Hence, the discussion will further delve into the two- and seven-equation model families.

#### 2.3.1 K-epsilon turbulence models

This family of turbulence models relates Reynolds stresses with mean flow quantities, as the Boussinesq approximation suggests, which led to Eq. (13).

(13) $$-\bar{\rho u_{i}^{\prime \prime }u_{j}^{\prime \prime }}=2\mu_{t}S_{\text{ij}}-\frac{2}{3}\rho k\delta_{\text{ij}}$$

$S_{\text{ij}}$ is the strain-rate tensor, k denotes the turbulent kinetic energy per unit of mass and $\mu_{t}$ is the turbulent viscosity (eddy viscosity). The standard k−ε model was originally published by Launder and Spalding [31,32], adding two transport equations: one for k and other for its rate of dissipation (ε). The eddy viscosity is the key feature in the two-equation models and is defined as Eq. (14) shows for the standard k-ε model.

(14) $$\mu_{t}=\rho C_{\mu }\frac{k^{2}}{\varepsilon }$$

The standard *k-ε* model is one of the most general tools for calculating turbulent flows, where several constants are considered (see Table 1). The constants of the model were estimated for common flow configuration such as cooling films, mixing layers, jets, confined and unconfined flows [5,14,15].

**Table 1:** Standard k−ε model constants.

$C_{1\varepsilon }$,	$C_{2\varepsilon }$,	$C_{3\varepsilon }$	$\sigma_{k}$	$\sigma_{\varepsilon }$
1.44	1.92	0.09	1.0	1.3

However, contradictory results have been reported in scientific literature. Mahmud et al. [33] conducted a sensitivity analysis of constants $C_{1\varepsilon }$ and $C_{2\varepsilon }$, for a lifted non-premixed turbulent free jet flame. The purpose of this analysis was to assess the effect of these model constants on the spreading rate of the jet. The $C_{1\varepsilon }$ value was varied within a range of 1.44–1.66 and $C_{2\varepsilon }$ was varied within a range of 1.87–1.92. It was found that the best overall model fit corresponds to the default constants values. Nevertheless, several authors argue about the capability of standard k−ε model for predicting the spreading rate, decay rate and length of the recirculation zone in planar, round and axisymmetric jets [9,12,34]. The issue was extensively addressed by Pope [35], several modifications were analyzed by the author. The analysis conducted by the author suggests the need for tuning model constants in the case of jets. Although there is a general understanding that a good balance between simplicity and model robustness is achieved when the model constant value $\left(C_{1\varepsilon }\right)$ is modified from 1.44 to 1.6 [34,36,37]. Additionally, it has been reported as a successful model improvement for Bluff-Body jet of non-premixed flame [38,39].

Several improvements have been made to the standard k−ε model. RNG *k-ε* is obtained by a statistical technique called Renormalization Group Theory. The model is derived from the standard k−ε, but includes an additional term in the dissipation rate of kinetic energy equation for suddenly strained flows. The effect of swirling motion is included, which is considered as a significant advantage over standard model. Prandtl number is computed by a sub-model, making the model capable of assessing heat or momentum diffusivity contribution to the fluctuations of the turbulent flow field [19,[40], [41], [42]]. Realizable k−ε model was developed by Shih et al. [43]. A new transport equation for kinetic energy dissipation was derived from the dynamic equation of the mean-square vorticity fluctuations at high Reynolds numbers. Additionally, an alternative turbulent viscosity model was formulated, which satisfies realizable condition of normal and shear stresses, ensuring the positivity of normal stresses and the Schwarz's inequality for shear stresses [19,43]. Realizable k−ε model performs notably better than the standard k-ε model in some flow conditions, including the round-jet anomaly showed by standard k−ε model. Some authors choose the realizable model over others k−ε models for high Reynolds number jets, even when swirling motion is important [44].

#### 2.3.2 K-omega turbulence models

The standard k−ω model used in the presented work is based on the Wilcox model [45]. The model is enhanced by modification for low Reynolds number effects, shear flow spreading and compressibility effects. Despite the decreasing freestream sensitivity of professional CFD codes regarding k−ω model, other authors point out that final solutions are still severely affected by freestream sensitivity [46]. The model has a strong empirical basis, derived from numerical DNS experiments, making it suitable for high Reynolds numbers in highly confined or near-wall flows. Additionally, it is part of the two-equation models family, where the transport equations represent turbulence kinetic energy (k) and specific dissipation rate (ratio of k and ε). Turbulent viscosity is obtained from Eq. (15), where $\alpha^{*}$ is the damping coefficient for correcting the turbulent viscosity at low Reynolds number.

(15) $$\mu_{t}=\alpha^{*}\frac{\rho k}{\omega }$$

Two new models, form the two-equation eddy-viscosity family, were developed by Menter [47]. The baseline (BSL) k−ω model addresses the well-known freestream sensitivity issue of Wilcox model. The BSL k−ω model combines the accuracy of Wilcox model near the walls with the freestream independency of the k−ε model in regions away from the walls. The standard k−ε model is transformed into k−ω formulation. Both models are simultaneously implemented but multiplied by a blending function, which selectively activates the k−ε model in the freestream region and deactivates k−ω. Despite enhancements made to the original Wilcox model, a substantial freestream sensitivity remains, partly due to the lack of accounting for shear stress transport by the model [19,48]. Shear-Stress Transport (SST) k−ω model includes all the refinements made by the BSL k−ω model and incorporates the shear stress transport in the turbulent viscosity model. This inclusion minimizes the overestimation of the turbulent viscosity in the free stream region. The SST model is suitable for a wide range of flow conditions, including adverse pressure gradient, airfoils and transonic shock waves [14,19,49]. However, it is not clear what specific advantages the SST model may provide over other turbulence models for axisymmetric jets.

The RANS modelling approach covers a wide range of basic flow configurations with reasonable accuracy. However, the turbulence models differ from each other in terms of robustness, near-wall treatment and interoperability [19,46,47]. The Generalized k−ω (GEKO) model aims to provide a single turbulence model, which would be flexible enough to satisfy a wide range of turbulent flow conditions [50]. The model has six parameters that can be calibrated to address physics and complexity of the domain [51]. Some authors argue about the calibration of $C_{\text{SEP}}$ and $C_{\text{JET}}$ parameters. GEKO k−ω model could provide similar results as the modified version of standard k−ε model in terms of spreading rate phenomena in an axisymmetric jet [19,51].

#### 2.3.3 Reynolds stress model

Reynolds stress models (RSM) or second-moment closure models are based on the original work of Launder et al. [52,53]. RSM are considered the most elaborate turbulent models, where turbulence isotropy is partially abandoned. Reynolds-Average Navier-Stokes equations are closed by solving a transport equation for Reynolds stress and another for the dissipation rate. RSM are particularly useful when turbulence isotropy is not a valid approximation of the turbulent flow state. However, due to the need to model the pressure-strain and dissipation-rate terms, under fairly isotropy assumption, similar assumptions are made as in the two-equation eddy-viscosity models [12,19].

## 3 Experimental and numerical setup

The experimental data used in this work is freely published at the International Workshop on Measurement and Computation of Turbulent Flames (TNF Workshop) [16]. The apparatus studied is a turbulent jet diffusion-flame. It consists of a cylindrical nozzle with a length of 350 mm and an internal diameter of 140 mm, along with an axially located tube with an internal diameter of 8 mm. The tube is used to supply a fuel mixture with an exit velocity of 42.2 m/s $\left(1.389∙10^{-3}kg/s\right)$, as shown in Fig. 1a and b. Dry air is supplied at the bottom of the flame with a velocity of 0.3 m/s $\left(3.853∙10^{-2}kg/s\right)$. As the height increases beyond x=300mm, the surrounding room air, which includes dust and humidity, reaches the flame contours. Further information about the burner can be found in the work presented by Barlow and Masri [17,18].

**Fig. 1:** a) DLR jet-flame test-facility [16], b) DLR-jet-flame geometry for the simulation.

Fuel and air were supplied at temperature of 293 K. The fuel has a volumetric composition of $33.2\%\;H_{2}$, $22.1\%\;{\text{CH}}_{4}$ and $44.7\%\;N_{2}$, which lead to a stoichiometric mixture fraction of 0.16. The ambient pressure, during the measurements, was 95300 Pa and the adiabatic flame temperature reached was of 2130 K [54]. Three experiments were performed: one at the German Aerospace Center (DLR), a second at Darmstadt University of Technology, and the third at Sandia National Laboratories, showing acceptable agreement among them. In general, more detailed information regarding the experimental data, the error sources and the uncertainties regarding measure techniques used can be found in TNF Workshop records and in the work of Barlow [16,54,55].

The simulations were carried out using the professional software ANSYS-Fluent. Table 2 shows the turbulence models assessed for the reacting turbulent jet-flow. All simulations began with a baseline 2D-axisymmetric mesh, followed by a mesh size scaling-up process to ensure results independence from the mesh size for all simulations. The experimental setup was recreated in an axisymmetric domain of 1.02 m in x direction and 0.19m in y direction. The fuel nozzle was geometrically modelled with 0.020 m of length, ensuring a fully developed flow at the exit plane of the fuel jet, as well as the cylindrical section for the supply of combustion air. The meshes were built by increasing the mesh density by a factor of five in the direction of the flame bottom and the axisymmetric axis. According to Masri et al. [18] and Meier [54], experimental data provides reasonable evidence that suggests a symmetrical behavior of the flame, making it possible to consider only half of the domain for the performed simulations. The meshes were assessed by means of two metrics: Orthogonal Quality and Cell Equiangle Skewness, obtaining an Orthogonal Quality close to one and a Cell Equiangle Skewness below to 0.01.

**Table 2:** Turbulence models assessed.

Turbulence model	Description
k−ε models	
Standard k−ε	Two-equation eddy-viscosity model
Realizable k−ε	Two-equation eddy-viscosity model
RNG k−ε	Two-equation eddy-viscosity model
Standard modified k−ε	Two-equation eddy-viscosity model
k−ω models	
Standard k−ω	Two-equation eddy-viscosity model
BSL k−ω	Two-equation eddy-viscosity model
GEKO k−ω	Two-equation eddy-viscosity model
SST k−ω	Two-equation eddy-viscosity model
Reynolds Stress models	
RSM-LPS	Five-equation RSM model (2D)
RSM-SO	Five-equation RSM model (2D)
RS-SBSL	Five-equation RSM model (2D)

The mesh independence analysis was performed considering up to three meshes for each turbulence model. Fig. 2 exhibits the mesh independence analysis for the standard modified k−ε model, where the axial velocity and temperature were studied at three locations (x=0.1m,x=0.3m and x=0.5m) of the combustor centerline. The solid lines correspond to the temperature values, and the dashed lines correspond to the axial velocity values, obtained after the simulations were carried out. Temperature and axial velocity values showed an asymptotic behavior between the second mesh (mesh #2, with 92,860 cells) and the third mesh (mesh #3, with 171,980 cells), as shown in Fig. 2. It can be considered that results are independent of the mesh size at mesh #2, as the third simulation showed no appreciable difference between results obtained from mesh #2 and mesh #3. Therefore, the second mesh (as shown in Fig. 3) was selected as the solution to be compared against experimental data. This choice allows us to save computational resources in post-processing and in future simulations. Similar analyses were carried out for other turbulence models, yielding similar results.

**Fig. 2:** Mesh independence analysis for k-ε standard modified version. Baseline (BL) mesh has 33780 cells, mesh 2 (M2) has 92860 cells and mesh 3 has 171980 cells.

**Fig. 3:** Mesh grading distribution of the meshed domain.

Simulations were carried out for a steady state condition and the pressure-velocity algorithm selected was SIMPLEC. It was established as the convergence criteria residuals for energy and radiation in the order of $1\times 10^{-9}$ and for the other magnitudes residuals on the order of $1\times 10^{-6}$. Additionally, mass and energy imbalance were assessed, yielding values in the order of $1\times 10^{-15}$.

## 4 Results and discussion

Simulation results were analyzed in terms of axial and radial velocity, temperature, mean mixture fraction, and species mass fraction data using the mean deviation from the experimental results, as shown in Eq. (16). $q_{\exp}$ represents each experimental measurement and q stands for the data obtained from simulation results.

(16) $$\text{MD}=\frac{\sum \left(\left|q_{\exp}-q\right|\right)}{\sum \left(\left|q_{\exp}\right|\right)}$$

Fig. 4 shows the mean deviation of axial velocity (*U*), radial velocity (*V*), mean mixture fraction (*ξ*), temperature (*T*) and major species mass fraction (YO_2_, YH_2_O, CO_2_ and CO). Fig. 5 shows the mean deviation of minor species mass fraction (YOH and YNO). The simulation results were categorized by turbulence model family (k−ε*,* k−ω and Reynolds Stress models), as shown in Table 2. The differences among each turbulence model family led authors to select the best turbulence model of each group for further analysis, which makes it possible to determine the optimal RANS turbulence modelling approach for the analyzed case. From Fig. 4, Fig. 5, it can be appreciated that standard modified k−ε model outperforms other k−ε models. The standard modified *k-ε* model showed the lowest mean deviation for the axial velocity, mean mixture fraction, temperature and profiles of species mass-fraction. However, it is worth noting that RNG k−ε the model performed slightly better than the standard modified *k-ε* model in terms of radial velocity. The results of k−ω models showed a similar performance among them, being standard k−ω slightly better than other k−ω models, which showed the lowest mean deviation for the axial velocity, major species and NO species mass fraction. Nevertheless, generalized k−ω (GEKO k−ω) performs better than the other k−ω models in terms of radial velocity deviation, while the BSL k−ω outperforms the other k−ω models in terms of OH mass fraction.

**Fig. 4:** Mean deviation of axial velocity (*U*), radial velocity (*V*), mean mixture fraction (*ξ*), Temperature (T) and major-species mass-fraction (YO_2_, YH_2_O, CO_2_, CO).

**Fig. 5:** Mean deviation of minor-species mass-fraction (YOH and YNO).

Among Reynolds-stress models, RSM-SBSL exhibits the best results fit to experimental measurements. According to Fig. 4, Fig. 5, the RSM-SBSL model showed the lowest mean deviation for axial velocity, mean mixture fraction, temperature, $O_{2}$ mass fraction, $H_{2}O$ mass fraction and ${\text{CO}}_{2}$ mass fraction. Meanwhile, RSM-LPS exhibited a lower mean deviation than RSM-SBSL for radial velocity, CO mass fraction and OH mass fraction. In general, mean deviation of all turbulence models showed that standard modified k−ε outperforms all analyzed turbulence models, except for radial velocity magnitude.

### 4.1 Flow field data analysis

The flow field variable (U,V), corresponding to each radial sample taken from the standard modified k−ε, Standard k−ω and RSM-SBSL models results are shown in Fig. 6, Fig. 7. It can be appreciated that all turbulence models can capture the shapes of each radial and axial velocity profiles.

**Fig. 6:** Axial velocity profiles for experimental data, standard modified k-ε (St. Mod. *k-ε*) model, standard *k-ω* model and Stress Baseline Reynolds-stress (SBSL-RS) model.

**Fig. 7:** Radial velocity profiles for experimental data (Exp), standard modified *k-ε* (St. Mod. *k-ε*), standard *k-ω* and Stress Baseline Reynolds-stress (SBSL-RS) model results.

Nevertheless, according to the data plotted on Fig. 8, standard modified k−ε fits better the experimental data than standard k−ω and RSM-SBSL for radial samples between x/d=5 to x/d=40. The k-ε model showed difficulties in representing flow field variables (U,V) near the fuel nozzle (x⁄d=1/8) and in the zone where radial velocity profiles exhibited a higher scattering behavior (x⁄d=60andx⁄d=80). In general, a high mean deviation of radial velocity is evidenced across all turbulence models, suggesting the inadequacy of both the two-equation eddy-viscosity model and the five-equation model in capturing the magnitude of such pronounced fluctuation patterns. This observation holds true from a quantitative perspective, emphasizing the limitations of these models in accurately representing the turbulent behavior.

**Fig. 8:** Mean deviation of radial samples for axial velocity (*U*, left side) and radial velocity (*V*, right side); for standard modified *k-ε* (St. Mod. *k-ε*), standard *k-ω* and Stress Baseline Reynolds-stress (RSM-SBSL) model results.

According to Pope and Shin et al. [9], an ideal plane jet and an axisymmetric jet spread linearly in the main flow direction. The flow is statistically two-dimensional and can be globally characterized by two quantities: centerline velocity $\left(U_{0}\left(x\right)\right)$ and half-width $y_{1/2}\left(x\right)$, respectively defined by Eq. (17) and Eq. (18).

(17) $$U_{0}=\left\langle U_{0}\left(x,0,0\right)\right\rangle$$

(18) $${\frac{1}{2}U}_{0}=\left\langle U_{0}\left(x,y_{1/2}\left(x\right),0\right)\right\rangle$$

Fig. 9 compares samples taken from experimental and computational results of the mean centerline velocity (left side) and the inverse of centerline velocity scaled-up by the mean jet velocity at exit nozzle plane (right side). The mean centerline velocity exhibits a larger deviation in comparation to experimental results for dimensionless axial distance below x/d=10, which corresponds to the developing zone of the jet [56]. The standard modified k−ε model showed a better performance than the other models in terms of mean centerline velocity for downstream distance above x/d=10. On the other hand, standard modified k−ε model shows the decay rate of centerline velocity in accordance with experimental data up to x/d=40. Meanwhile, for x/d=60 and x/d=80, the centerline velocity exhibits a slower decay rate than the experimental data. This leads to an overestimation of mean axial velocity for such radial profiles, as can be appreciated in Fig. 6.

**Fig. 9:** Mean centerline velocity (right side) and the inverse of scaled-up centerline velocity (right side). In the figure, experimental data (Exp); standard modified k-ε model (St. Mod. k-ε), standard k-ω model and Stress Baseline Reynolds-stress model (RSM-SBSL).

Fig. 10 shows the behavior of turbulent kinetic energy dissipation at the combustor centerline. The curves for the RSM-SBSL model and the standard modified k−ε model exhibit a similar shape and trend. However, the curve for the standard k−ω model exhibits a different trend compared to the other two models, especially between x/d=10 and x/d=60. The peak of maximum kinetic energy dissipation, at the combustor centerline, occurs at the same sample location (x/d=20) for the standard modified *k-ε* model and RSM-SBSL model. However, the values are quite different, the peak of kinetic energy dissipation for the RSM-SBSL model being higher than for the standard modified k−ε model.

**Fig. 10:** Dissipation of turbulent kinetic energy at the combustion centerline (left side) and zoom in of turbulent kinetic energy dissipation up to x/d=10. In the figure, standard modified *k-ε model* (St. Mod. *k-ε*), standard *k-ω* model and Stress Baseline Reynolds-stress model (RSM-SBSL).

The similarity of the *ε* magnitude, in terms of the shape of the curves and trend, for the standard modified k-ε model and the Stress Baseline Reynolds-stress model is reflected on the axial velocity profiles (Fig. 6) and on the centerline axial velocity (Fig. 9). It turns out that even a minor variation in the dissipation of turbulent kinetic energy has a significant impact on the values of the axial velocity profile. The distribution of the kinetic energy dissipation rate for standard k−ω was quite different than the results shown by the standard modified k−ε model and RSM-SBSL model. The peak of ε magnitude shift from x/d=20 to x/d=40, for the k−ω model. Quantitatively speaking, the magnitude of ε peak was lower for this model than the other turbulence models. The impact of the poor representation of ε magnitude, shown by the standard k−ω models, is reflected in the mean velocity at the combustion centerline, as Fig. 9 shown. In the same zone (x/d=20, x/d=40 and x/d=60), where ε magnitude has shown similarities between k−ε model and Reynolds-stress model, axial velocity profiles (Fig. 6) obtained by these models fit experimental data better than standard k−ω model. However, at the zone close to the fuel nozzle, the standard k−ω outperforms the other turbulence models. A zoom-in of Fig. 10 (left side), corresponding to the locations between x/d=1/8 to x/d=10, is shown in Fig. 10 (right side). The behavior of ε magnitude in terms of shape and trend is very similar for all turbulence models, the main differences between each model's results are quantitative, with the highest values of ε magnitude for standard modified k−ε model and the lowest values for the RSM-SBSL model. As result, mean deviations of axial and radial velocity profiles at the location x/d=1/8 are lower for the standard k−ω model than the other models (see Fig. 8).

Fig. 11 shows the streamlines, colored by the dissipation rate of turbulent kinetic energy, in the zone corresponding to 5 mm downstream from the fuel nozzle up to 45 mm in the streamwise direction of the combustion zone. It could be appreciated the shear layer formed between fuel and air stream, with the values of ε being even higher at the shear layer zone than at the combustor centerline.

**Fig. 11:** Streamlines colored by the dissipation rate of turbulent kinetic energy for standard modified k−ε, standard k−ω and Stress Baseline Reynolds-stress (RSM-SBSL) model results; y-direction and x-direction of the graphic in millimeters.

The standard modified k−ε model shown the higher values of turbulent kinetic energy dissipation and the RSM-SBSL model the lowest values. According to Fig. 6, Fig. 7, it can be appreciated that axial and radial velocity profiles obtained from standard k−ω model at x/d=1/8 zone fit better experimental measurements. However, downstream axial and radial velocity profiles, between x/d=5 to x/d=60, showed that standard modified k−ε model fits better experimental data than the other turbulence models.

The jet's Reynolds number for the analyzed case study is 22,800 and according to Pope [9] self-similarity region for turbulent jet with $\text{Re}>10^{4}$ begin at dimensionless streamwise distance of x/d>30. Additionally, the author points out that experimental observations suggest that all dimensionless profiles collapse into a single curve. Fig. 12 shown that dimensionless Jet's self-similar velocity profiles for standard k−ω suggests the exclusion of the profiles at x/d=10 from the self-similar region, which corresponds to the experimental observations. However, the velocity profile at x/d=20 is out of Jet's self-similar region and results obtained by the standard k−ω model suggest the oppositive. The experimental data suggests a decay rate of centerline velocity in the self-similarity region of the jet as $U_{0}∼x^{-1}$. The standard k−ω model exhibited a decay rate of centerline velocity within the range of the experimental data. Nevertheless, the standard modified k−ε model and RSM-SBSL model showed that centerline velocity decay as $U_{0}∼x^{-0.88}$ and $U_{0}∼1/x^{-1.1}$, respectively.

**Fig. 12:** Dimensionless axial velocity profile, x/d=10 (*◊*), x/d=20 (*⁎*), x/d=40 (*Δ*), x/d=60 (*×*) and x/d=80 (***○***), for experimental measurements (Exp); standard modified k−ε (St. Mod. k−ε), standard k−ω and Stress Baseline Reynolds-stress (RSM-SBSL) model results.

### 4.2 Species and temperature data analysis

Fig. 13 compares the profiles of the mean mixture fraction, temperature, and major species mass fraction between experimental measurements and the samples obtained from computational results. A qualitative analysis of the results suggests that the computational results manage to represent the profile shapes of major species mass fraction, temperature, and mean mixture fraction. In general, the standard modified k−ε model exhibits better performance in terms of mean mixture fraction, temperature and species mass fraction, except for the NO mass fraction. In Table 3, the color pattern uses red for the highest mean deviation, yellow for intermediate values, and green for the lowest mean deviation across all turbulence models for each magnitude. The mean deviation data show that standard modified k−ε model outperforms the standard k−ω model and RSM-SBSL model in the region between x/d≥10 to x/d≤60. However, close to the fuel nozzle and at x/d=80, RSM-SBSL model and standard k−ω model exhibit a better fit to the experimental data than the standard modified k−ε model. At x/d=5, RSM-SBSL model has shown the lowest mean deviation for the mean mixture fraction, temperature, $O_{2}$, $H_{2}O$ and ${\text{CO}}_{2}$ mass fractions, except for NO mass fraction.

**Fig. 13:** Profiles of mean mixture fraction, temperature and major species (legend: solid line for standard modified k−ε model, dashed line for standard k−ω model and dotdash line for RSM-SBSL model).

**Table 3:** Mean deviation of radial samples for the mean mixture fraction, temperature and species mass fraction for the computational results of standard modified *k-ε* (St. Mod. *k-ε*), standard *k-ω* and Stress Baseline Reynolds-stress (RSM-SBSL) model results.

The mean mixture fraction is an important scalar quantity in non-premixed combustion models as it provides a measure of the mixing process between fuel and oxidizer species. As a transport variable, the mean mixture fraction is significantly affected by the performance of the turbulence model. Table 3 highlights RSM-SBSL model results as the best in terms of mean mixture fraction for radial samples taken at x/d=5.The low intensity of the kinetic energy dissipation, between x/d=0 to x/d=5, is consistent with the good agreement of experimental data and RSM-SBSL model results, in terms of mean fixture fraction. It sems that the low kinetic energy dissipation shown by the results of RSM-SBSL model contributed to the ability of the model to accurately represent the mixing process in the zone close to fuel nozzle.

Additionally, the radial samples taken of RSM-SBSL model results at x/d=80 shown the lowest mean deviation for the mean mixture fraction, temperature and species mass fraction, except for NO mass fraction. Fig. 14 shows the mean mixture fraction contours with the axial velocity streamlines for the three analyzed turbulence models. For the RSM-SBSL model, streamlines at x/d=80, collapses faster onto the shear layer of the jet than for the other turbulence models.

**Fig. 14:** Local mean mixture fraction with axial velocity streamlines for the standard modified *k-ε* (St. Mod. *k-ε*), standard *k-ω* and Stress Baseline Reynolds-stress (RSM-SBSL) model results.

Fig. 15 shows a photograph of the experiment temperature field and the temperature contour of the computational results. The temperature distribution over the computational domain has shown some differences between the results of the turbulence models and the picture of the experiment Results from the RSM-SBSL model have shown the lowest temperature mean deviation for radial samples taken at x/d=5, x/d=10 and x/d=80. Meanwhile, at x/d=20, x/d=40 and x/d=60, the standard modified k−ε model results have shown the lowest temperature deviation. In the experiment, the adiabatic flame temperature reaches a value of 2130 K [17], and computational results have shown values of 1907 K for the standard modified *k-ε* model, 1911 K for the standard *k-ω* and 1856 K for the RSM-SBSL model.

**Fig. 15:** Photograph of the DLR jet flame [16] (Exp) and temperature contour for the computational results of the standard modified *k-ε* (St. Mod. *k-ε*) model, standard *k-ω* model and Stress Baseline Reynolds-stress (RSM-SBSL) model.

The performance of the standard modified k−ε model in the zone between x/d≥10 to x/d≤60, concerning flow field variables and mean mixture fraction, has resulted in more accurate outcomes from the turbulence-chemistry interaction model. In general, mean mixture fraction is more influenced by turbulence models than chemistry-turbulence interaction model (turbulent combustion model). On the other hand, temperature and species mass fraction are influenced by the turbulent combustion model as well as by the turbulence model.

Fig. 16 illustrates the profiles of OH and NO species mass fractions. Qualitatively, the profiles depicted in Fig. 16 fairly capture the shapes observed in the experimental data profiles. However, quantitative speaking the results for NO mass fraction notably deviate from the experimental values. The high mean deviation of NO mass fraction, as indicated in Table 3, is especially pronounced for the RSM-SBSL model compared to the other turbulence models. Other authors have reported the incapability of steady diffusion flamelet model to accurately estimates NOx species formation route [57,58]. There are several factors that affect the computation of NOx species by the turbulent combustion models, but one of the most important is related to the wide difference in kinetic time scale respect to other species formation and the assumption of fast chemistry for all species formation route.

**Fig. 16:** Profile of minor species mass-fraction (OH and NO); legend: solid line for the standard modified *k-ε* model, dashed line for the standard *k-ω* model and dotdash line for the RSM-SBSL model.

## 5 Conclusions

Eleven Reynolds-Average Navier-Stokes turbulence models were tested for the simulation of a CH_4_/H_2_/N_2_-Air reacting jet. Mean deviations compared to available experimental data were quantified for quantities of interest such as axial velocity, radial velocity, mean mixture fraction, temperature, major and minor species mass fraction, to assess the quality of the turbulence models. Standard modified k−ε, standard k−ω and RSM-SBSL model were found the most reliable options. Nevertheless, the spreading rate is disturbed for axisymmetric jet simulations carried out. The standard modified k−ε model has exhibited the best results, but some slightly underestimation of combustor centerline velocity decay-rate remains for the streamwise direction x/d>60. In the zone close to the fuel nozzle, the results from the standard k−ω have shown a lower mean deviation for the axial and radial velocity, showing the x/d=10 velocity profile better self-similarity conditions than the profiles obtained from the other turbulence models. The data obtained from the computational results suggest that the mean mixture fraction is strongly influenced by the performance of the turbulence model. Meanwhile, temperature and species mass fraction are affected by the turbulence model performance and the turbulence-chemistry interaction model. Additionally, the overestimation of NOx species mass fraction by the steady diffusion flamelet is still an issue and the result from this model should be carefully considered.

## Data availability

The data will be made available on request.

## Additional information

No additional information is available regarding this paper.

## CRediT authorship contribution statement

**Yaniel Garcia Lovella:** Writing – review & editing, Writing – original draft, Visualization, Methodology. **Idalberto Herrera Moya:** Writing – review & editing, Visualization, Supervision, Methodology, Conceptualization. **Jeevan Jayasuriya:** Writing – review & editing, Supervision, Methodology, Conceptualization. **Julien Blondeau:** Writing – review & editing, Supervision, Methodology, Conceptualization.

## Declaration of competing interest

The authors declare that they have no known competing financial interests or personal relationships that could have appeared to influence the work reported in this paper.
